This article has been retracted.

# circFAT1(e2) Promotes Papillary Thyroid Cancer Proliferation, Migration, and Invasion via the miRNA-873/ZEB1 Axis

**DOI:** 10.1155/2020/1459368

**Published:** 2020-10-19

**Authors:** Jiazhe Liu, Hongchang Li, Chuanchao Wei, Junbin Ding, Jingfeng Lu, Gaofeng Pan, Anwei Mao

**Affiliations:** Minhang Hospital, Fudan University, 170 Xin-Song Road, Shanghai 201199, China

## Abstract

Circular RNAs (circRNAs) play an extremely important regulatory role in the occurrence and development of various malignant tumors including papillary thyroid cancer (PTC). circFAT1(e2) is a new type of circRNA derived from exon 2 of the FAT1 gene, which is distributed in the cytoplasm and nucleus of PTC cells. However, so far, the role of circFAT1(e2) in PTC is still unclear. In this study, circFAT1(e2) was found to be highly expressed in PTC cell lines and tissues. circFAT1(e2) knockdown suppressed PTC cell growth, migration, and invasion. Also, circFAT1(e2) acted as a sponge for potential microRNAs (miRNAs) to modulate cancer progression. A potential miRNA target was discovered to be miR-873 which was targeted by circFAT1(e2) in PTC. The dual-luciferase assay conducted later also confirmed that there was indeed a direct interaction between circFAT1(e2) and miR-873. This study also confirmed that circFAT1(e2) inhibited the miR-873 expression and thus promoted the ZEB1 expression, thus affecting the proliferation, metastasis, and invasion of PTC cells. In conclusion, the results of this study indicated that circFAT1(e2) played a carcinogenic role by targeting the miR-873/ZEB1 axis to promote PTC invasion and metastasis, which might become a potential novel target for therapy of PTC.

## 1. Introduction

Circular RNA (circRNA) is a special type of alternative splicing (called reverse splicing) that produces a specifically and covalently closed-loop structural RNA [1]. Recently, several studies have shown that circRNAs are differentially expressed in various diseases [2], including cancer, atherosclerotic vascular diseases, and neurological diseases. This may suggest that circRNA could play a potential regulatory role in the progression of some diseases [3]. For example, circRNAs could bind to RNA polymerase II in a variety of ways to form complexes that could regulate the activity of RNA polymerase II and then affect parental gene transcription thereby [4]. According to the study of Abdelmohsen et al., circular PABPN1 (polyadenylate-binding nuclear protein 1) and HuR (human antigen R) can be extensively bound to form the HuR-circRNA complex, which competitively inhibits the binding of HuR and PABPN1 mRNA, leading to a decrease in the PABPN1 translation, thus disrupting the normal metabolism of cells [5]. Studies have also shown that the binding of circRNA UBAP2 to miR-143 can abolish the inhibition of Bcl-2 and the caspase apoptosis pathway [6].

Papillary thyroid cancer (PTC) is one of the most popular cancers in females [7]. The global incidence of PTC ranks 9th among all cancers [8]. The factors contributing to the progression of PTC are unclear. Despite several pieces of evidence have indicated that obesity, smoking, hormonal exposure, and certain environmental contaminants may be related to PTC [9–12], the only risk factor validated in PTC is ionizing radiation [13]. Therefore, there was an urgent need to identify novel regulators for the understanding of molecular mechanisms and biomarkers for the prognosis of this cancer [14]. circRNA plays an important role in thyroid cancer. For example, circRNA circZFR promotes the expression of C8orf4 by acting as a sponge on miR-1261 and facilitates the growth of PTC cells [15]. circRNA circRNA_102171 regulates CTNNBIP1-dependent activation through the *β*-catenin pathway to promote PTC progression [16]. circRNA circ-ITCH inhibits the progression of PTC via the miR-22-3p/CBL/*β*-catenin pathway.

circFAT1(e2) is a type of circRNA derived from exon 2 of the FAT1 gene and mainly exists in the cytoplasm of gastric cancer cells. Studies have shown that circFAT1(e2) is reduced in tissues and cell lines in gastric cancer (GC). Furthermore, mechanism analysis indicated overexpressed circFAT1(e2) could hinder the proliferation and metastasis of GC cells [17]. In this study, we focused on the role of circFAT1(e2) in PTC, and this finding might promote the prognosis and treatment of PTC.

## 2. Materials and Methods

### 2.1. Cell Lines and Cell Culture

The human thyroid normal cell line Nthy-ori 3-1 and the PTC cell lines CAL-62, TPC-1, and K1 were all from ATCC (Manassas, VA, USA). All cells were placed in an incubator at 37°C containing 5% CO_2_ and cultured using DMEM (BI, Israel) supplemented with 10% FBS (Invitrogen).

### 2.2. Cell Fractionation Assay

The cell fractionation assay was conducted according to a previous report [18]. Approximately 3 × 10^6^ cells were grown on 10 cm dishes (Corning), trypsinised, washed in cold 1x PBS, and centrifuged (1200 rpm, 5 min). Pellets were lysed in 1 mL hypotonic lysis buffer (10 mM HEPES pH 7.9, 10 mM KCl, 1.5 mM MgCl2, 1 mM *β*-mercaptoethanol, 0.075% NP-40, 1x murine RNase inhibitor, 1x protease/phosphatase inhibitor cocktails, Roche) and incubated for 15 min at 4°C with rotation. Nuclei were pelleted by centrifugation (1200 rpm, 4°C) for 15 min. The cytoplasm was collected from the supernatant. Nuclei were washed three times in 800 *μ*L PBS and collected as the pelleted nuclear fraction. Fractionated cytoplasmic and nuclear lysates were confirmed by localization of GAPDH and histone 3.1, respectively.

### 2.3. Dual-Luciferase Reporter Assay

For the sake of constructing luciferase reporter vectors, the whole circFAT1(e2) or the 3′UTR fragment of ZEB1 that contained the expected latent binding sites was cloned into the pmiR-RB-REPORT™ luciferase reporter vector (RiboBio, Guangzhou, China) at the Xhol and Notl sites; the same was true for the construction of a mutant sequence of circFAT1(e2) or ZEB1 at the 3′UTR.

For the dual-luciferase activity assay, we applied Lipofectamine 2000 (Invitrogen) to cotransfect each construct with marked miRNAs (RiboBio) in PTC cells for 48 h. The Dual-Luciferase Reporter Assay System (Promega, WI, USA) was performed under the instructions of the manufacturer. Besides, the BioTek Synergy HTX multimode reader was used to obtain the luminescent signals, and the luciferase activities were displayed according to the relative hRluc/hluc ratio.

### 2.4. qRT-PCR

Total RNA was extracted with the TRIzol reagent (Invitrogen, USA). For circRNA and mRNA, the reverse transcription of total RNA to cDNA was performed by reverse transcriptase (Vazyme, Nanjing, China). And then, we conducted qPCR with a SYBR Green PCR Kit (Vazyme, Nanjing, China). The fluorescence quantitative PCR instrument was QuantStudio™ 6 Flex manufactured by Thermo Fisher Scientific (USA). Besides, Sangon (Shanghai, China) was used to construct all the primer sequences. GAPDH was selected as the reference gene for circRNA and mRNA, and the internal control for miRNA was set as U6. We also used the 2^-*ΔΔ*Ct^ method to quantify the gene expression.

### 2.5. CCK-8 Assay

According to the instruction of the manufacturer (Dojindo Laboratories, Kumamoto, Japan), the proliferative ability of PTC cells was assessed with a CCK-8 assay. Next, we plated the CAL-62 and TPC-1 cells (1 × 10^3^ cell/well) in 96-well plates, treated them with 10 *μ*L of CCK-8 solution for 2 hours, and then analyzed spectrophotometrically at 450 nm by an automatic microplate reader.

### 2.6. Transwell Migration and Invasion Assays

The transwell chamber (Corning, NY, USA) was used to conduct the assays of cell migration and invasion. It could be directly used for migration assay, or with Matrigel mix (BD Biosciences, San Jose, CA, USA) for invasion assay. After incubation for 48 h, we used cotton swabs to scrape the cells which settled on the upper layers of the transwell chambers and fixed the cells settled on the lower surfaces. Next, we observed the number of cells in the transwell chambers under a fluorescent inverted microscope and took a photo.

### 2.7. Statistical Analysis

We used the form average value ± SD to present a continuous variable. We used one-way ANOVA [19] and Student's *t*-test [20] for multiple comparisons. All the analyses were performed in the software GraphPad Prism, v5.0 (GraphPad, La Jolla, CA, USA). In this paper, a significant difference was identified by a *p* value < 0.05.

## 3. Results

### 3.1. circFAT1(e2) Increased Abnormally in PTC Samples and Cell Lines

Compared with Nthy-ori 3-1 cells, the expression levels of circFAT1(e2) in K1, TPC-1, and CAL-62 cells were increased by onefold, twofold, and fourfold, respectively (Figure 1(a)). Furthermore, the circFAT1(e2) expression levels in 12 pairs of PTC tissues were also detected using qRT-PCR. The results indicated that the circFAT1(e2) expression in PTC tissues was higher than that in matched normal tissues remarkably (Figure 1(b)).

### 3.2. Silencing circFAT1(e2) Suppressed PTC Cell Proliferation

To determine the biological roles of circFAT1(e2) in TC, we firstly detected its subcellular location in CAL-62 and TPC-1 cells. Our results indicated that circFAT1(e2) is mainly located in the cytoplasm of TC cells (Figure 2(c)). Meanwhile, nuclear-located U6 and cytoplasm-located GAPDH were also detected as a positive control (Figures 2(a) and 2(b)). Next, we knocked down the expression levels of circFAT1(e2) in TC cells using a specific siRNA targeting of this circRNA (Figures 2(d) and 2(f)). In order to search the function of circFAT1(e2) knockdown on cell proliferation in TC cells, CCK-8 assays were performed. Our results showed that the proliferation rate of cells with si-circFAT1(e2) was remarkably downregulated compared to the control group in both CAL-62 (Figure 2(e)) and TPC-1 cells (Figure 2(g)).

### 3.3. circFAT1(e2) Suppressed PTC Cell Metastasis In Vitro after Knockdown

Furthermore, we then tested whether circFAT1(e2) would affect the metastatic abilities of PTC cells. Migration assay results indicated that circFAT1(e2) knockdown remarkably weakened the migratory capability of CAL-62 (Figures 3(a) and 3(b)) and TPC-1 cells (Figures 3(c) and 3(d)). Besides, we detected the invasion ability of PTC cells by estimating the penetration of cells through Matrigel in a transwell chamber. As illustrated in Figure 4, we found that circFAT1(e2) knockdown inhibited cell invasion. The numbers of invading cells were, respectively, decreased by 80 percent and 85 percent in CAL-62 (Figures 4(a) and 4(b)) and TPC-1 (Figures 4(c) and 4(d)) cells transfected with si-circFAT1(e2) compared with the negative control group. Altogether, these results reveal that circFAT1(e2) is a positive regulator of TC metastasis.

### 3.4. circFAT1(e2) Served as a Sponge of miR-873 to Promote ZEB1

Previous studies have shown that circRNA could serve as sponges for miRNAs. In this study, we proposed that circFAT1(e2) might also serve as a miRNA sponge in TC. circFAT1(e2) is mainly located in the cytoplasm of TC cells. circFAT1(e2) may regulate the expression of target proteins at the posttranscriptional level, indicating that circFAT1(e2) may be the ceRNA of miRNAs. To test this hypothesis, we used miRanda (https://www.microrna.org/microrna/home.do) to predict the potential interaction between miRNAs and circFAT1(e2)1. We found that circFAT1(e2) and miR-873 had binding sites. Using HumanTargetScan, ZEB1 was predicted by bioinformatics as a potential target of miR-873 (http://www.targetscan.org/cgi-bin/targetscan/vert_71/). Previous studies have found that miR-873 is involved in the disease by targeting ZEB1 progress [21, 22]. ZEB1 was reported to be an oncogene in human cancers. qRT-PCR assay indicated that circFAT1(e2) knockdown significantly suppressed the expression levels of ZEB1 in both TPC-1 and CAL-62 (Figures 5(a) and 5(b)).

In order to further validate these findings, we detected the expression levels of circFAT1(e2) and ZEB1 after overexpressing miR-873 in PTC cells and found that overexpression of miR-873 remarkably suppressed the RNA levels of circFAT1(e2) and ZEB1 in TC cells (Figures 5(c)–5(f)). Dual-luciferase assays were performed to verify whether miR-873 could straightly interact with circFAT1(e2) and ZEB1. Luciferase reporters were cotransfected with miR-873 into PTC cells. The pmiR-RB-Report vector containing 3′-UTR regions of ZEB1 or circFAT1(e2) cotransfected with miR-873 mimic significantly reduced the Renilla/firefly ratio in contrast to the control vector (Figures 5(g) and 5(i)). However, overexpression of miR-873 did not significantly influence the luciferase activity of the pmiR-RB-Report vector, which contained 3′-UTR-mut regions of ZEB1 or circFAT1(e2)-mut (Figures 5(h) and 5(j)). These results indicated that miR-873 could directly target circFAT1(e2) and ZEB1.

## 4. Discussion

In this study, circFAT1(e2) was found to be higher in papillary thyroid tumors and cell lines than that in normal thyroid tissues and cells. Interestingly, the downregulation of circFAT1(e2) modulated miRNA-873/ZEB1 signaling pathways. More importantly, circFAT1(e2) knockdown inhibited some physiological functions of PTC cells.

Many studies also indicated that circRNA played a crucial role in multiple types of human cancers, such as breast cancer, liver cancer, gastric cancer, and thyroid cancer. For instance, in Wei et al.'s study, it is showed that circZFR contributes to the growth of PTC cells by the miR-1261/C8orf4 axis [15]. By using the microarray analysis of circRNA in thyroid cancer, 98 circRNAs were found to be dysregulated. It was also found that circRNA-100395 had a significant potential for interaction with cancer-associated miRNAs [23]. Wang et al. revealed that circ-ITCH could inhibit the progression of PTC by regulating miR-22-3p/CBL/*β*-catenin cascade [24]. While it was unclear how circFAT1(e2) functions in PTC. This study showed elevated levels of circFAT1 (e2) in PTC. And it displayed that circFAT1(e2) promoted the development of PTC cells by affecting proliferation, invasion, and migration. The results in our study also suggested that circFAT1(e2) played a carcinogenic role in thyroid cancer, suggesting that circFAT1(e2) might be a potential therapeutic target.

In gastric cancer (GC), a novel circRNA circFAT1(e2) has been identified. circFAT1(e2) is significantly downregulated in GC tissue and is related to the overall survival rate of GC patients. circFAT1(e2) is distributed in the cytoplasm and nucleus of GC cells. circFAT1(e2) in the nucleus can directly interact with Y-box-binding protein 1 (YBX1) and inhibit its function. circFAT1 (e2) in the cytoplasm exerts a tumor suppressor effect by regulating the miR-548g/RUNX1 axis. Moreover, this study also demonstrates that overexpressed circFAT1(e2) induces the proliferation, migration, and invasion of GC cells, and it plays a tumor-suppressive role in GC [17]. Through our research, circFAT1(e2) is upregulated in PTC cells and tissues and may participate in cell proliferation, cell metastasis, cell invasion, and other biological processes. Also, we proved that the knockdown of circFAT1(e2) could inhibit the expression of ZEB1. miR-873 overexpression strongly suppressed the expression levels of ZEB1 and circFAT1(e2). Luciferase assay showed that miR-873 could reduce the activity of pmiR-RB-Report vector containing 3′-UTR regions of ZEB1 or circFAT1(e2). These results demonstrated that both ZEB1 and circFAT1(e2) were the direct targets of miR-873.

It has been demonstrated that miR-873 played different roles in different cancers [25]. It has been identified as an oncogene in lung adenocarcinoma [26], however, as a suppressor in breast cancer, ovarian cancer, and glioblastoma [27]. In glioma cells, overexpression of miR-873 leads to a decrease in Bcl-2, which in turn inhibits cell proliferation, cell metastasis, and cell invasion [28, 29]. In breast cancer cells, miR-873 not only depresses breast cancer cell proliferation but also enhances tamoxifen resistance [30]. Similarly, miR-873 has been shown to bind to IGF2BP1 in glioblastoma cells and depress the growth and metastasis of glioblastoma cells [31]. The functions of miR-873 in different cancer types could be different relying on the particular cellular environment. Consistently, it was revealed that miR-873 was downregulated in PTC cells according to our qRT-PCR results. ZEB1 is a transcription factor known for its ability to induce EMT carcinogenesis, which plays a role in cells through various mechanisms including Wnt, NF-*κ*B, and miRNAs [32]. In breast cancer cells, the transfection of miR-873 mimics decreased ZEB1 expression. ZEB1 can act as a transcriptional activator to activate YAP1 target genes, including the expression of AXL, CTGF, and CYR61, and also as a transcriptional repressor to inhibit the expression of the target gene (E-cadherin) consistently [33]. This study also confirmed that circFAT1(e2) inhibited the miR-873 expression and thus promoted the ZEB1 expression, thus affecting the proliferation, metastasis, and invasion of PTC cells.

In conclusion, we have proved that circFAT1(e2) promotes the tumorigenesis and invasiveness of PTC. It participates in the regulation of PTC by competitively binding with miR-873 and upregulating the expression of its target gene ZEB1. These findings suggest that the circFAT1(e2)-miR-873-ZEB1 axis may be a promising target for the prognosis and therapy of PTC.

## Figures and Tables

**Figure 1:** circFAT1(e2) increased abnormally in PTC samples and cells. (a) The circFAT1(e2) was more expressed in PTC cells. (b) PTC tissues had higher expression level of circFAT1(e2). ^∗^*p* < 0.05, ^∗∗^*p* < 0.01, and ^∗∗∗^*p* < 0.001.

**Figure 2:** Silencing circFAT1(e2) suppressed PTC cell proliferation. (a–c) circFAT1(e2) mainly located in the cytoplasm of TC cells. The efficiency of circFAT1(e2) knockdown was detected by qRT-PCR in CAL-62 (d) and TPC-1 (f) cells. CCK-8 experiments showed that circFAT1(e2) knockdown attenuated the proliferation capacity of CAL-62 (e) and TPC-1 (g) cells. ^∗^*p* < 0.05, ^∗∗^*p* < 0.01, and ^∗∗∗^*p* < 0.001.

**Figure 3:** circFAT1(e2) knockdown remarkably weakened the migratory capability of CAL-62 (a, b) and TPC-1 (c, d) cells. (a) Representative images of transwell migration assays in CAL-62 cells (scale bar, 45 *μ*m). (b) The quantification of transwell migration assays in CAL-62 cell. (c) Representative images of transwell migration assays in TPC-1 cells (scale bar, 45 *μ*m). (d) The quantification of transwell migration assays in TPC-1 cell. ^∗^*p* < 0.05, ^∗∗^*p* < 0.01, and ^∗∗∗^*p* < 0.001.

**Figure 4:** circFAT1(e2) silenced inhibited invasive capability of CAL-62 (a, b) and TPC-1 (c, d) cells. (a) Representative images of transwell invasion assays in CAL-62 cells (scale bar, 45 *μ*m). (b) The quantification of transwell invasion assays in CAL-62 cell. (c) Representative images of transwell invasion assays in TPC-1 cells (scale bar, 45 *μ*m). (d) The quantification of transwell invasion assays in TPC-1 cell. ^∗^*p* < 0.05, ^∗∗^*p* < 0.01, and ^∗∗∗^*p* < 0.001.

**Figure 5:** circFAT1(e2) served as a sponge of miR-873 to augment ZEB1. ZEB1 expression levels were lower in TPC-1 (a) and CAL-62 (b) cells with circFAT1(e2) knockdown by qRT-PCR. TPC-1 (c, e) and CAL-62 (d, f) cells transfected with miR-873 had less expression of circFAT1(e2), ZEB1. The luciferase activities of circFAT1(e2) and ZEB1 were measured in TPC-1 (g, i) and CAL-62 (h, j) cells transfected miR-873 mimics or miR-NC with dual-luciferase reporter assay. ^∗^*p* < 0.05, ^∗∗^*p* < 0.01, and ^∗∗∗^*p* < 0.001.

## Data Availability

The datasets used and/or analyzed during the current study are available from the corresponding author on reasonable request.
